The article "Deep Integration of Physical Health Education Based on Intelligent Communication Technology" was retracted in 2023. Reasons: suspected computer-generated content; unreliable results or conclusions; concerns about the data; concerns about the results or conclusions.

# Deep Integration of Physical Health Education Based on Intelligent Communication Technology

**DOI:** 10.1155/2021/4323043

**Published:** 2021-09-15

**Authors:** Min Liu, Jianjun Bu

**Affiliations:** Shanxi University, Taiyuan, China

## Abstract

In recent years, intelligent medical communication technology has developed rapidly, and the advancement of hardware technology has accelerated the development of software technology. Physical exercise breaks the limits of all aspects of the human body and requires scientific and reliable information. Industrial cameras realize collection and high-resolution image processing functions and use artificial intelligence to create conditions for collecting scientific data. With the powerful driving force of artificial intelligence, it is believed that physical education will develop to a new height. The intellectualization of physical education makes people expect that it will also bring some inevitable problems, but as long as we continue to overcome and improve, we believe that artificial intelligence will better serve physical education and benefit mankind. Artificial intelligence is the current trend of social development. This paper takes physical education as a breakthrough point to discuss the application of artificial intelligence in physical education. This paper uses the grey GM prediction model and questionnaire survey method to build an online education platform and develop an effective education model, which can integrate the country's best educational resources and reduce time and space constraints. Providing a relaxing learning environment for education, one can learn anytime, anywhere. In a typical physical education system, the average self-efficacy score is converted from 20.48 points to 68.37 points, and the average self-score of physical education in the integrated artificial intelligence environment is converted from 30.25 points to 75.54 points. The data show that the quality of education has greatly improved.

## 1. Introduction

### 1.1. Background and Significance

The concept of artificial intelligence (AI) was formally proposed at the Dartmouth Conference in 1956. It belongs to a major field of computer science and is known as one of the world's third largest technologies. Professor Jeavons, an expert at Stanford University in the United States, once defined artificial intelligence as follows: “Artificial intelligence is the field of knowledge. It is a way of expressing knowledge, but also a way of acquiring and using knowledge.” [1] Dr. Summerfield C. from the Massachusetts Institute of Technology in the United States believes that “artificial intelligence is the study of how computers perform intelligent tasks that only humans can perform.” [2] Artificial intelligence can recognize and deal with language, images, in-depth study, and so on, at this stage, artificial intelligence and human intelligence are likely to trigger simple thinking similar to the human mind in the process of simulating the creation of human conscience and thought, but in the future, it may even surpass human intelligence in some aspects. We must pay attention to the problems brought about by the development and application of artificial intelligence and constantly seek solutions to facilitate the entry of artificial intelligence into work and life. Therefore, the importance of this research theme lies in the ability to understand the self-efficacy of comprehensive sports through the analysis of the self-efficacy of sports students and the investigation and research on the distribution of future sports. Self-efficacy theory and many studies have found that when individuals face methods and challenges to perform specific tasks, the behavior of sports students will be affected by the degree of self-efficacy. Individuals with higher self-efficacy are more likely to try to complete specific tasks than individuals with lower self-efficacy [3, 4].

### 1.2. Related Work

Chen M. said that we are currently developing advanced computer and application technology, which is our computer and application technology aimed at improving the performance and reducing costs and supporting the latest applications more effectively in the network environment [5]. The development of computer and application technology is a long-term process. Generally speaking, computer technology has been committed to independent innovation and has made satisfactory breakthroughs in some technologies and applications. According to the existing applications, these technologies and applications closely follow the mainstream of international computer technology [6, 7]. Paper et al. believed that multimedia education can be used to improve students' interest in learning and learning efficiency [8]. This will help solve the key and difficult points in education. It has contributed to the realization of proper coordination and coordinated training [9]. The implementation of multimedia education should be combined with traditional education, pay attention to improve the quality of teachers, choose appropriate teaching methods, and timely collect information about the effect of education and focus on it [10], but their research is not accurate enough. The deep integration of physical education based on artificial intelligence technology has far exceeded their research.

### 1.3. Main Content

The research methods of this article include the literature research method, interdisciplinary research method, grey GM prediction model method, expert interview method, questionnaire survey method, and other research methods. According to the development and popularization of artificial intelligence in today's social life, the research on the combination of artificial intelligence and sports has been triggered. The research status and application of artificial intelligence in physical education and teaching are discussed and summarized, including the application of artificial intelligence technology in sports and the application in physical education.

The innovation of this article is to describe the value of artificial intelligence technology applied to physical education, which is explained separately from a macro- and microperspective. Reverse thinking, that is, the current limitations of artificial intelligence technology and physical education, illustrates that a good combination of the two cannot mature in a short period of time. It explains the trend of artificial intelligence technology in the development of physical education. The angle is summarized and judged based on the authors' research.

## 2. Deep Integration of Physical Education Based on Artificial Intelligence Technology

### 2.1. Grey GM Prediction Model

The user model was constructed by using education profile data and training strategy data, and the recommendation model was established by using the coordinated filtering recommendation algorithm. It also evaluates the physical strength and drive of the coach based on the practice results, adds the video and image data results from the sports education process and other data from the education process to the personal profile as the movement record, and updates the user model to improve the quality of education.

Grey system theory extracts useful information by generating and decomposing known information. In particular, it is difficult to lack the space for appropriate elements, the operating mechanism is not yet clear, and the information system is not enough to establish a clear relationship. The GM(1, 1) model is the key to grey prediction. This is a single-layer differential equation model for predictor variables. This discrete time response function is almost exponential. The modeling method of creating GM(1, 1) is as follows.

The original data series contains *K* items, where *X* represents nonnegative original time series data. The AGO method is used to establish *X*(1), and (*K*)=∑_*n*=1_^*k*^*X*^(0)^(*n*),  *k*=1,2,3,…, *n*, is obtained:

(1) $$\begin{array}{c} \frac{\text{d}x^{\left(1\right)}}{\text{d}t}+ax^{\left(1\right)}=b. \end{array}$$

It is the original form of the GM(1, 1) model. The original form of the GM(1, 1) model is essentially a difference equation. *k* is the time point, *a* is the development coefficient, and *b* is the grey effect. The value of *a* and *b* can be estimated by applying the least square method.

(2) $$\begin{array}{c} \hat{a}=\left[\begin{array}{c} a\\ b \end{array}\right]={\left(B^{T}B\right)}^{-1}B^{T}Y_{N}. \end{array}$$

### 2.2. Expert Interview Method

According to the requirements of this topic, interviews with relevant professionals, scholars, and sports workers will be conducted via e-mail or telephone. With the development of network technology applications, listen to the opinions of experts on some of the issues and opinions discussed in this article. This article listened to the opinions of university sports experts and teachers and provided a basis for summarizing the main problems of using network technology in university sports. Understand the reality of establishing a national sports university network, establishing a national sports school network, and developing university sports network courses.

### 2.3. Theoretical Analysis Method

This article first briefly introduces the application background of home network technology in college physical education and introduces and analyzes the current situation of the domestic and international network technology on college physical education and the needs of college physical education. On the basis of system analysis, it is necessary to be familiar with sports-related network skills and design and implement training courses for testing and analysis.

## 3. Comparative Experiment on the Deep Integration of Physical Education Based on Artificial Intelligence Technology

Due to the uneven distribution of educational resources in China, high-quality educational resources are usually concentrated in first-tier cities. Therefore, the demand for quality education resources in cities below the first tier is very high. At the same time, in addition to the increasing pressure of learning, the working population is under increasing competitive pressure. As the pressure of competition increases, the demand for learning and growth of the labor force also increases.

### 3.1. Choice of Teaching Method

According to the survey, the most commonly used teaching methods for college physical education tutors are lectures (accounting for 85%), teaching methods (accounting for 75%), and theoretical research methods (accounting for 43.3%). Seminars, lectures, and other methods are not often used, and the proportion is too small. According to a large number of literature studies, it is learned that college physical education students have gradually lost interest in traditional teaching methods and have become more interested in seminars and other methods. The survey data are shown in Table 1.

Sports majors need updated knowledge. They are not interested in boring theoretical training and are more focused on practical training. Interest is a good teacher for students to learn. Therefore, teachers of college physical education students need to select network technology reasonably and apply it to the educational combination to transform boring pure theoretical knowledge into vivid teaching methods.

### 3.2. Role Positioning

The role of college physical education teachers is as follows: facilitator and instructor of student learning, facilitator of student physical and mental development, participant of school construction and management, collaborator, and learner and innovator of scientific research. Compared with traditional courses, the content of college physical education students using the internet to learn courses is designed by teachers and students through an interactive process, rather than textbooks written by experts or scholars. For this type of online education, university teachers must act as information consultants, emotional advocates for participant learning, and organizers of course training. The survey data are shown in Figure 1.

The application of artificial intelligence technology in university sports has exacerbated the weakening of university teachers. The traditional university physical education model has always dominated the leadership or dominant position of university teachers. College physical education students study through the internet. The characteristics of this course are different from those of regular courses. Its content is not a textbook edited by experts or scholars, but an interactive process composed of teachers and students using artificial intelligence technology.

## 4. Data Analysis of Survey Results

After research and extensive literature review and extensive distribution of conclusions, the application of artificial intelligence technology has had a greater impact on the philosophy, concepts, learning attitudes, and learning environment of the university's graduate school of physical education, and it has changed the concept of university physical education teachers. When it comes to the teacher-student relationship, it can have a big impact. In terms of organizing and managing college graduates, artificial intelligence technology started early and formed a certain model, as shown in Table 2.

In today's universities, the current training model of physical education students restricts the development of the subjective initiative of the instructors, and the training of practical skills is ignored in some learning processes of physical education students. When promoting this model, college physical education teachers underestimated the educational effects of educational institutions.  Figure 2 shows the impact of artificial intelligence technology on sports students in colleges and universities.

The learning philosophy of physical education students in colleges and universities is different from that of high school students or ordinary college students. Through investigations, it is found that the learning philosophy of physical education students does not stop at the acquisition of knowledge, but is reflected in the development of personality. Among them, learning to be a person, learning to learn, and learning to do is accounted for the proportions of them all exceed 50%. The data are shown in Figure 3.

Analyzing the above data, we draw the following conclusions: in the network environment, sports graduates can acquire knowledge and information faster and have more available space. This requires continuous learning and absorbing new knowledge, and artificial intelligence technology can continuously change learning concepts and improve learning capabilities to keep up with the continuous updates of science and technology. The results also show that the use of artificial intelligence technology in university education has a significant impact on the learning philosophy of sports students. Existing sports students always think that there is no need to improve their professional level, focus on theoretical research, or ignore theoretical research and blindly emphasize practice. In fact, practice and theory do not match; this concept is wrong. The introduction of artificial intelligence technology is very helpful to improve the professional or theoretical level of sports majors.

## 5. Conclusions

Artificial intelligence has brought great changes to human development since its birth. Many aspects of the current social life have been affected by it, and physical education will inevitably join the trend. Traditional physical education, in the background of increasingly sophisticated artificial intelligence technology, the use of computers and big data analysis, and other science and technology, will give people a brand new experience. Through a thorough elaboration and understanding of the subject, the intervention of a new technology may cause disturbance to the existing system, including positive effects and many problems, but the key lies in the original intention of the person mastering the technology, the ability to use the technology, and the ability to solve the problem. In the field of physical education, the introduction of artificial intelligence and its branches has produced positive effects, but the problems it has brought must be solved. For example, as an AI coach who makes educational programs scientifically, it expands the scope and depth of information collection. The AI-assisted physical education is a shock to the traditional coaches. Intelligent algorithms recommend educational programs that not only enhance user stickability but also may lead to unpredictable risks or “information cocoon room” for users; smart sensors collect user feedback to provide real data for later improvement of the accuracy of education programs, but at the same time, there is a risk of privacy user disclosure. In the face of this challenge, educators and coaches must learn to embrace and apply new technologies. Privacy protection mechanism should be set for artificial intelligence education equipment to obtain information. Develop and improve the intelligence of robots by mastering hidden intelligence; teachers improve their skills when facing impact; when the algorithm is popular, we should pay more attention to the value of humans as the subject.

The application of artificial intelligence technology in my country is still in its infancy. Motion video computer vision research needs to enhance the motion video data standard, the formulation of the motion image data standard, and the standardized algorithm for video image processing. Expertise in image processing equipment is also the key to success. Intelligent video technology still has a long way to go to improve the understanding of hardware devices, establish sports video image standards, and improve video tracking and processing algorithms. The application of enhanced video technology in sports videos is the only way to develop sports videos. Artificial intelligence technology also affects physical education. In real life, with the help of artificial intelligence technology, it is already possible to learn sports theory knowledge and relatively basic sports support. Experts in artificial intelligence theory at home and abroad have proven that future machines can produce knowledge, emotion, understanding, and even imagination of human intelligence. All of these artificial intelligence technologies are applied to the mature physical education field, providing athletes with great convenience and efficiency. In fact, the development speed of artificial intelligence technology in the education field is actually faster than expected.

## Figures and Tables

**Figure 1:** The role of college physical education teachers in teaching.

**Figure 2:** Influence of the network technology on sports graduate students in colleges and universities.

**Figure 3:** Statistics table of the learning philosophy of postgraduates in physical education.

**Table 1:** Selection of commonly used teaching methods for college physical education teachers.

	Frequently used		Occasionally used		Uncommonly used	
	*N*	%	*N*	%	*N*	%
Lecture	51	85.00	9	15.00	0	0.00
Taught	45	75.00	10	10.00	5	8.33
Theoretical research	26	43.33	26	46.33	8	13.34
Seminar	2	3.33	9	15.00	49	81.66
Lecture style	3	5.00	12	20.00	45	75.00

**Table 2:** The influence of the network technology on physical education graduate students in colleges and universities.

	Great influence		Big influence		Influential		Small influence		No effect	
	*N*	%	*N*	%	*N*	%	*N*	%	*N*	%
Learning philosophy	37	41.11	28	31.11	18	20.00	7	7.78	0	0.00
Learning attitude	42	46.67	23	25.60	18	20.00	7	7.78	0	0.00
Learning environment	41	45.56	19	21.11	17	18.90	13	14.40	0	0.00
Learning ability	26	28.90	25	27.80	26	28.90	13	14.40	0	0.00
Learning path	26	28.90	24	26.70	20	22.22	10	11.11	0	0.00

## Data Availability

The data underlying the results presented in this study are available within the article.
